The article "A simple and rapid method for detection of Goose Parvovirus in the field by loop-mediated isothermal amplification" was published in 2010. Journal: Virol J.

# A simple and rapid method for detection of *Goose Parvovirus *in the field by loop-mediated isothermal amplification

**DOI:** 10.1186/1743-422X-7-14

**Published:** 2010-01-21

**Authors:** Yang JinLong, Yang Rui, Cheng AnChun, Wang MingShu, Fu LiZhi, Yang SongQuan, Zhang SuHui, Yang Liu, Xu ZhiYong

**Affiliations:** 1 Chongqing Academy of Animal Science, Chongqing 402460, Chongqing, China; 2 Avian Diseases Research Center, College of Veterinary Medicine of Sichuan Agricultural University, Yaan 625014, Sichuan Province, China; 3 Key Laboratory of Animal Diseases and Human Health of Sichuan Province, Yaan 625014, Sichuan Province, China; 4 College of Animal Sciences, Henan Institute of Science and Technology, Xinxiang 453003, Henan Province, China

## Abstract

**Background:**

Goose parvovirus (GPV) is a *Dependovirus *associated with latent infection and mortality in geese. Currently, in a worldwide scale, GPV severely affects geese production. The objective of this study is to develop a loop-mediated isothermal amplification (LAMP) method for the sensitive, rapid, and inexpensive detection of GPV in the field.

**Results:**

A set of six specific primers was designed by targeting the GPV VP3 DNA. With *Bst *DNA polymerase large fragment, the target DNA could be amplified at 65°C as early as 20 min of incubation in a simple water bath. A positive reaction was identified through the detection of the LAMP product by color change visible to the naked eye. The detection limit of the assay was 28 copies/μl of plasmid pVP3, and with equal sensitivity and specificity to fluorescent quantitative real-time PCR (FQ-PCR).

**Conclusions:**

The high sensitivity, specificity, and simplicity, as well as the high throughput, make this method suitable for specific detection of GPV infection in both field conditions and laboratory settings. The utilization of complicated equipment and conduct of technical training on the GPV LAMP were not necessary.

## Background

Goose parvovirus (GPV) is a well known causative agent of Gosling plague (GP), an acute, contagious, and fatal disease referred to as Derzsy's disease [1]. GPV has been formally classified as a member of the genus *Dependovirus *under the family, *Parvoviridae *[2]. It was first described as a clinical entity by Fang [3]. In the realm of research, GPV has attracted much attention owing to tremendous economic loss for countries engaged in industrialized goose production; the virus infection has spread rapidly worldwide, resulting in high rates of morbidity and mortality [1,4-6].

Several detection methods have been developed for identifying GPV, such as agar-gel diffusion precipitin test, virus neutralization (VN) assay, enzyme-linked immunosorbent assay (ELISA) [5], qualitative PCR [7,8], and fluorescent quantitative real-time PCR (FQ-PCR) [9]. All are effective and accurate in detecting the virus infection in laboratory settings, but they require the use of expensive equipment and are laborious and time-consuming. Thus, these methods are considered unfavorable for use on a large-scale basis. In contrast, a more preferred detection method would be one that is not only speedy and sensitive, but also simple and economical during practical applications [10].

Recently, a loop-mediated isothermal amplification (LAMP) reaction was developed as an alternative method to meet the abovementioned requirements. The LAMP method allows the whole reaction process, including denaturing, to proceed at a constant temperature by incubating the reagents in a simple incubator. As a specific nucleic acid amplification method, it can easily perform and amplify nucleic acid at isothermal conditions (i.e., 60-65°C) within 1 h of incubation [11-13]. LAMP reaction requires four or six primers based on six or eight distinct regions of the target DNA, hence allowing high degree of specificity during viral detection. The presence of amplified products can be detected at a short time. By the end of the reaction, the presence or absence of the target DNA can be judged visually by the appearance of a white precipitate of magnesium pyrophosphate, or a green color of the solution stained by SYBR green I. The presence of multiple bands of LAMP reaction products in agarose gel electrophoresis indicates a mixture composed of stem-loop DNAs with various sizes of stem and cauliflower-like structures having multiple loops, which is induced by alternately annealing inverted repeats of the target sequence in the same strand [11,14]. In addition, the LAMP method does not require any special reagent or sophisticated temperature control device. Since it only needs simple equipment, cost-effective genetic tests can be easily achieved. Both simple detection and real-time detection of the reaction are deemed possible http://loopamp.eiken.co.jp/e/index.html. Specifically, the LAMP method has already been applied in the specific detection of animal viruses, such as *hepatitis B virus *[15], *Japanese encephalitis viral *[16], and *H9 avian influenza virus *[17]. However, to the best of our knowledge, no study has yet used the technique to detect GPV. In this study, we report the development of LAMP assay for the specific, rapid, and sensitive detection of GPV in infected goslings.

## Results

### Optimized LAMP reaction

LAMP reaction was performed using plasmid (pVP3) DNA as template in order to determine optimal temperature and time of reaction. The amplicons were formed at 61, 62, 63, 64, and 65°C and the clearest product was detected at 65°C (Fig. 1A). Thus, 65°C was used as the optimal temperature for the succeeding assays. Meanwhile, LAMP products were also detected as early as 20 min at 65°C (Fig. 1B). Although well-formed bands in the system could be detected as early as 20 min, reaction time was optimized and set at 40 min to ensure positive detection of templates with lower concentration.

**Figure 1:** **Determination of the optimal temperature and time of LAMP**. (A) Determination of the optimal temperature. Lane M: DL-2000 marker; lanes 1: -, negative control; 2--7: LAMP carried out at 60, 61, 62, 63, 64 and 65°C, respectively. (B) Determination of the optimal time. lane M, DL-2000 marker; lanes 1: -, negative control; 2-7, LAMP carried out for 10, 20, 30, 40, 50 and 60 min, respectively. All the products were electrophoresed on a 2% agarose gels and stained with ethidium bromide.

### Specificity of the LAMP assay

The specificity of LAMP and FQ-PCR was tested using templates extracted from GPV and other viruses. Only GPV showed a positive reaction; no DNA band was observed from the other seven animal pathogens (Fig. 2). Results of FQ-PCR (data not shown) correlated well with the LAMP method [9], indicating that LAMP is as specific as FQ-PCR for GPV detection.

**Figure 2:** **Agarose gel illustrating the specificity of the GPV-LAMP assay among different species**. The reaction was carried out at 65°C for 40 min. Lane M: DL-2000 marker; lanes 1 and 2: GPV-CHv and pVP3 as positive control; lane 3:-, negative control; 4: ADV; 5: CPV; 6: PPV; 7: NDV; 8: *Pasteurella multocida *(5: A); 9: *Salmonella enteritidis *(No. 50338); 10: *Escherichia coli *(O78).

### Sensitivity of LAMP assay

The detection limit of LAMP using plasmid DNA was set at 28 copies/μl (Fig. 3). In comparison with the detection limit of FQ-PCR (date not shown) [9], LAMP was observed to similarly sensitive to the FQ-PCR system.

**Figure 3:** **Sensitivities of LAMP for detection of plasmid pVP3**. Lane M: DL-2000 marker; 1--12, reaction carried out using 10-fold serial dilutions of plasmid (pVP3) DNA (2.8 × 10^11 ^copies/μl). 1: 2.8 × 10^0^, 2: 2.8 × 10^1^, 3: 2.8 × 10^2^, 4: 2.8 × 10^3^, 5: 2.8 × 10^4^, 6: 2.8 × 10^5^, 7: 2.8 × 10^6^, 8: 2.8 × 10^7^, 9: 2.8 × 10^8^, 10: 2.8 × 10^9^, 11: 2.8 × 10^10^, 12: 2.8 × 10^11 ^copies/μl, respectively; lane 13:+, positive control; lane 14:-, negative control. All the products were electrophoresed on a 2% agarose gels and stained with ethidium bromide.

### Detection of LAMP products by naked eye observation

LAMP products could also be detected with the naked eye by observing white turbidity in the reaction mixture (Fig. 4A) or by color change of the solution stained by SYBR Green I (Fig. 4B). As shown by Fig. 4A, white turbidity could be observed from products of the reaction with 2.8 × 10^2 ^to 2.8 × 10^11 ^copies/μl of plasmid, but not from the negative control and the 2.8 × 10^0 ^to 2.8 × 10^1 ^copies/μl. In Fig. 4B, after the addition of 1 μl of diluted SYBR Green I to the reaction tube, the color of the LAMP reaction solution changed from orange to green in the 2.8 × 10^1 ^to 2.8 × 10^11 ^copies/μl of plasmid template DNA, while no color change was observed in the 2.8 × 10^0 ^copies/μl and in the negative control. These show that the LAMP detection limit could be set at 2.8 × 10^2 ^copies/μl to observe white turbidity, and 2.8 × 10^1 ^copies/μl to observe color change in the reaction solution. The color observation method is 10 times more sensitive than the white turbidity observation method.

**Figure 4:** **Detection of LAMP products by observing white turbidity and color of the reaction mixture**. (A) shows white turbidity of the reaction mixture by magnesium pyrophosphate; (B) shows color (green) of the reaction mixture after addition of SYBR Green I. N, negative control; 1--12, reaction carried out using 10-fold serial dilutions of plasmid (pVP3) DNA (2.8 × 1011 copies/μl). 1: 2.8 × 10^0^, 2: 2.8 × 10^1^, 3: 2.8 × 10^2^, 4: 2.8 × 10^3^, 5: 2.8 × 10^4^, 6: 2.8 × 10^5^, 7; 2.8 × 10^6^, 8: 2.8 × 10^7^, 9: 2.8 × 10^8^, 10: 2.8 × 10^9^, 11: 2.8 × 10^10^, 12: 2.8 × 10^11 ^copies/μl, respectively; 13:+, positive control.

### Application of the LAMP assay for detection of GPV infection in goslings

Optimal LAMP assay was evaluated by analyzing GPV infected gosling tissues. DNA extracted by the tissue boiling method gave rise to a typical ladder pattern, as shown in Fig. 5. GPV was positively detected in infected gosling spleen, kidney, and liver (Fig. 5). Thirty clinical cases with suspected GPV infections were investigated using both the LAMP assay and FQ-PCR. Twenty-one of the 30 samples were tested positive, while nine were negative, based on FQ-PCR and LAMP, indicating well concordance between the two methods (data not shown) when performed on gosling tissues.

**Figure 5:** **Detection of GPV in infected gosling tissues by LAMP**. lane M: DL-2000 marker; 1, negative control 2, positive control; 3, spleen; 4, kidney; 5, liver.

## Discussion

China currently holds the largest waterfowl population in the world with a production industry characterized by increased expansion and rapid development in the past decades [18]. However, infectious diseases represent the biggest obstacle to the successful development of this business. GPV is one of the most serious viral pathogens in the goose industry. Since prevention and early detection are presently the most logical strategies for virus control, the most effective way of controlling the disease would be by conducting routine screening of this virus [19]. However, thus far, no practical (e.g., simple and rapid) method is available for the specific diagnosis of GPV in field conditions.

The use of the LAMP reaction has been successfully established in diagnosing viral infections in human and animals [15-17]. In the present study, a LAMP protocol was developed as a rapid and simple detection tool for the specific diagnosis of GPV. No cross-reaction with three other related virus (i.e., Aleutian disease virus or ADV; canine parvovirus or CPV; and porcine parvovirus or PPV) and four other unrelated animal pathogens (i.e., Newcastle disease virus or NDV; *Pasteurella multocida*, 5:A; *Salmonella enteritidis*, No. 50338; and *Escherichia coli*, O78) was observed in the FQ-PCR and LAMP detection. The specificity of LAMP was not affected by the presence of non-target genomic DNA in the reaction mixture, a characteristic highly desirable in the development of a diagnostic system [11]. The LAMP method used for GPV detection was observed to be highly sensitive, and other studies have shown that detection of target DNA by LAMP, compared to FQ-PCR, was equally sensitive [20,21], a finding confirmed by our results. In other words, the specificity and the detection limit of the LAMP assay are equal with FQ-PCR for detecting GPV.

The optimal condition for detecting GPV by LAMP was determined to be at 65°C for 40 min. However, it was also observed that the LAMP products could be detected as early as 20 min. In addition, there were fewer operational steps for the LAMP assay than for conventional PCR and FQ-PCR assays, and expensive equipment is not necessary to obtain high level precision [22]. LAMP is a more rapid method for detecting animal virus, as compared to either the PCR or FQ-PCR method, which separately need at least 2-3 h [23] to complete. In practice, the time required for diagnosis is considered to be crucial for farm and hatchery management in goslings breeding. Hence, its rapid characteristic makes it a useful tool for GPV diagnosis.

Real-time monitoring of LAMP amplification can be accomplished through agarose gel analysis. LAMP amplicons revealed a ladder-like pattern in contrast to a single band as observed in PCR (Fig. 1). This is due to the cauliflower-like structures with multiple loops formed by annealing between alternately inverted repeats of the target in the same strand [24].

Furthermore, gel electrophoresis is not needed because the LAMP method synthesizes a large amount of DNA where the products can be detected by simple turbidity or fluorescence [17]. Thus, expensive equipment is not necessary to obtain high level precision--one equivalent to or greater than those of other PCR techniques. In order to facilitate the field application of the LAMP assay, the monitoring of amplification can be accomplished with naked eye inspection through visual fluorescence. LAMP is a simple and effective method that utilize SYBR Green I for visual inspection of amplification products less the required use of gel electrophoresis and staining with ethidium bromide. The visual inspection for amplification products could be performed by observing color change following the addition of 1 μl of SYBR Green I to the tube. The orange color of the dye will change into green under natural light with positive amplification. For cases with no amplification, the orange color of the dye is retained [24]. The sensitivity of inspection by white turbidity was inferior to the use of SYBR Green I or the electrophoresis method (Fig. 4A) because tenfold more copies of template DNA were needed to obtain a positive reaction, as compared to SYBR Green I or the electrophoresis method. The eye inspection method was simple and rapid, but offered difficulty in detecting quantitative amplification. Yet, the eye inspection method could facilitate the application of LAMP, especially as a field test [10].

Our final goal is to establish a simple and rapid diagnostic method for GPV in field applications. Using LAMP assay, the only equipment needed is a water bath, which is used for both the DNA preparation and nucleic acid amplification. With no complicated equipment and the necessary technical training, LAMP assay is considered very simple and easy to operate. LAMP can be operated in most situations where rapid diagnosis is required such as under field conditions. In particular, LAMP is capable of detecting the presence of pathogenic agents faster than PCR, even on the first day of fever when the amount of GPV copy number is very low, due to its higher sensitivity and given the detection limit of about 28 copies. Earlier detection of infection implies earlier treatment and return to good health [24]. Thus, we recommend that this technique be applied routinely in order to conduct timely survey on GPV infection in goose farming. In doing so, the virus-carrying goslings can be identified during the early stages of infection; countermeasures can be devised even before the infection becomes epizootic.

## Conclusions

In conclusion, the LAMP protocol described in this study represents a new inexpensive, sensitive, specific, and rapid protocol for the detection of GPV. Compared to FQ-PCR and other assays, LAMP does not require strict reaction conditions or complicated technical operation or special equipment. Instead, this method requires only a water bath. This protocol provides an important diagnostic tool for the detection of GPV infection in both laboratory and field settings.

## Materials and methods

### Goslings, tissues, virus, DNA, and standard plasmid DNA templates preparation

Goslings, tissues, virus, and standard plasmid DNA templates were prepared as described by Yang [9]. To obtain crude DNA by tissue boiling method, approximately 100 mg of tissue from goslings was homogenized in 1000 μl of 1% SDS in 100 mM Tris-HCl (pH 8.0), boiled for 10 min, and centrifuged at 10,000 g for 5 min. The supernatant was transferred to a new tube and used immediately [10].

### Design of LAMP primers

A set of six species-specific LAMP primers was designed to target the GPV sequence (GenBank: U25749). Briefly, the highly conserved VP3 region of the GPV gene was selected and used as the LAMP target. LAMP primers were designed using the PrimerExplorer V4 software program http://primerexplorer.jp as following: Forward outer primer (F3); Backward outer (B3); Forward inner primer (FIP); Backward inner (BIP); Loop Forward (LF); and Loop Backward (LB). The sequences of the primers and their locations are shown in Table 1 and Fig. 6.

**Figure 6:** **Schematic diagram of primers' sequences and positions for LAMP**. (A). Nucleotide sequence of partial GPV VP3 used to design inner and outer primers for LAMP. The nucleotide sequences and the positions used to design the primers. (B). A schematic diagram showing the positions at which the primers attach for amplification of the target gene.

**Table 1:** The primers used for LAMP

Primer	Type	5'pos	3'pos	Length	Sequence
F3	Forward outer	1209	1228	20-nt	5'-ggtttggcagaacagggata-3'
B3	Backward outer	1406	1425	20-nt	5'-gcccgtagagtactgggtta -3'
FIP	Forward inner (F1c +F2)			40-mer(F1c:22-nt, F2:18-nt)	5'-ggccaaatcctccgagattcgg-cagggacctattggggca -3'
BIP	Backward inner(B1c +B2)			40-mer (B1c:20-nt, B2:20-nt)	5'-caatccaccaccgcaggtgt-ccacttctggtgcacgtatt -3'
LF	Loop Forward	1259	1283	25-nt	5'-TGGAATTTACCATCAGTCTTCGGTA-3'
LB	Loop Backward	1339	1362	24	5'-ATCAAGAATACACCAGTGCCTGCA-3'

### LAMP reaction

LAMP was carried out in a 25 μl total reaction volume containing 0.2 μM each of F3 and B3, 0.8 μM each of FIP and BIP, 0.4 μM each of the LF and LB primers, 1.0 mM dNTPs, 1 M betaine (Sigma), 25 mM Tris-HCl (pH8.8), 10 mM KCl, 10 mM (NH_4_)_2_SO_4_, 5 mM MgSO_4_, 0.1% Triton X-100, eight units of the *Bst *DNA polymerase large fragment (New England Biolabs), and 1.0 μl of template DNA. Reaction time was optimized by incubating the mixture for 10, 20, 30, 40, 50, and 60 min at a pre-determined temperature (65°C), while the reaction temperature was optimized by incubating the mixture at 60, 61, 62, 63, 64, and 65°C at a pre-determined time (60 min). The reaction was terminated via heating at 80°C for 5 min. LAMP products (3 μl) were electrophoresed on 2% agarose gels and stained with ethidium bromide to determine the optimal conditions.

### Observation of LAMP products by naked eye

Amplified DNA in the LAMP reaction causes white turbidity due to the accumulation of magnesium pyrophosphate, a by-product of the reaction. LAMP amplicons in the reaction tube were directly detected by the naked eye by adding 1.0 μl of a thousand-fold-diluted original SYBR Green I (Molecular Probes Inc.) to the tube, and by observing the color of the solution. The solution changed from light orange to green in the presence of LAMP amplicons, while it remained light orange in the absence of amplification. Prior to the addition of SYBR Green I, white turbidity of the reaction mixture by magnesium pyrophosphate was also inspected. The reaction mixture (3 μl) was analyzed by 2% agarose gel electrophoresis, and then ethidium bromide-stained and visualized.

### FQ-PCR detection

Detection was performed as described by Yang [9].

### Specificity of LAMP assay

The specificity of the assay was tested by using templates from pVP3, GPV-CHv, and several other pathogens, including ADV, CPV, PPV, NDV, *Pasteurella multocida *(5:A), *Salmonella enteritidis *(No. 50338), and *Escherichia coli *(O78) (Key Laboratory of Animal Diseases and Human Health of Sichuan Province). FQ-PCR was carried out as control assay.

### Sensitivity of the LAMP assay

The detection limits of the assay were evaluated using tenfold serial dilutions of plasmid (pVP3). The plasmid DNA (2.8 × 10^11^copies/μl) was serially diluted tenfold, and 1 μl of each dilution was used as templates for the LAMP reaction. Reaction was performed at 65°C for 60 min and compared with the FQ-PCR assay.

### Application of LAMP to detect GPV infection in gosling tissues

In order to evaluate the optimal LAMP assays for the detection of GPV, total DNA from tissues (spleen, kidney, and liver) of experimental infected goslings was extracted via the boiling method, as described above, for 72 h post-infection. Gosling tissues were analyzed by LAMP and FQ-PCR to detect the virus infection.

Thirty suspected clinical cases previously collected from natural outbreaks of the disease were selected for LAMP test. FQ-PCR was carried out as control assay.

## Competing interests

The authors declare that they have no competing interests.

## Authors' contributions

JY and YR carried out most of the experiments and wrote the manuscript, and should be considered as first authors. AC and MW critically revised the manuscript and the experiment design. LF, YS, ZS, XZ and YL helped with the experiment. All of the authors read and approved the final version of the manuscript.
